# Combination effect of cold atmospheric plasma with green synthesized zero-valent iron nanoparticles in the treatment of melanoma cancer model

**DOI:** 10.1371/journal.pone.0279120

**Published:** 2022-12-19

**Authors:** Zahra Yazdani, Pourya Biparva, Alireza Rafiei, Mostafa Kardan, Seyedehniaz Hadavi

**Affiliations:** 1 Department of Immunology, Molecular and Cell Biology Research Center, School of Medicine, Mazandaran University of Medical Sciences, Sari, Iran; 2 Student Research Committee, Mazandaran University of Medical Sciences, Sari, Iran; 3 Department of Basic Sciences, Faculty of Animal Science and Fisheries, Sari Agricultural Sciences and Natural Resources University, Sari, Iran; 4 Department of Atomic and Molecular Physics, Faculty of Basic Sciences, University of Mazandaran, Babolsar, Iran; 5 Plasma Technology Research Center, Faculty of Basic Sciences, University of Mazandaran, Babolsar, Iran; Kwangwoon University, REPUBLIC OF KOREA

## Abstract

Green synthesized zero-valent iron nanoparticles (nZVI) have high potential in cancer therapy. Cold atmospheric plasma (CAP) is also an emerging biomedical technique that has great potential to cure cancer. Therefore, the combined effect of CAP and nZVI might be promising in treatment of cancer. In this study, we evaluated the combined effect of CAP and nZVI on the metabolic activity of the surviving cells and induction of apoptosis in malignant melanoma in comparison with normal cells. Therefore, the effect of various time exposure of CAP radiation, different doses of nZVI, and the combined effect of CAP and nZVI were evaluated on the viability of malignant melanoma cells (B16-F10) and normal fibroblast cells (L929) at 24 h after treatment using MTT assay. Then, the effect of appropriate doses of each treatment on apoptosis was evaluated by fluorescence microscopy and flow cytometry with Annexin/PI staining. In addition, the expression of BAX, BCL2 and Caspase 3 (CASP3) was also assayed. The results showed although the combined effect of CAP and nZVI significantly showed cytotoxic effects and apoptotic activity on cancer cells, this treatment had no more effective compared to CAP or nZVI alone. In addition, evaluation of gene expression showed that combination therapy didn’t improve expression of apoptotic genes in comparison with CAP or nZVI. In conclusion, combined treatment of CAP and nZVI does not seem to be able to improve the effect of monotherapy of CAP or nZVI. It may be due to the resistance of cancer cells to high ROS uptake or the accumulation of saturated ROS in cells, which prevents the intensification of apoptosis.

## Introduction

Cutaneous melanoma is the 12^th^ most common cancer in the world with an incidence rate of 3.0 per 100,000 [1, 2]. The prevalence of this cancer is increasing in both industrial and non-industrial countries. Therefore, the development of new anticancer strategies is needed [2]. Cold atmospheric plasma (CAP) is a new promising therapy in various types of cancers such as cutaneous melanoma. CAP is an ionized gas near room temperature, consisting of reactive oxygen (ROS), reactive nitrogen (RNS) species, and optical emission in the UV range that is produced at atmospheric pressure [3–5]. This modality is used for wound healing, tissue regeneration, and surface sterilization [6, 7]. The current evidence shows that the effect of CAP on cancer cells is higher than that of normal cells due to the increase in the level of ROS and RNS in cancer cells, which will eventually increase their death by inducing apoptosis in vitro [8–10].

Apart from the anticancer activity of CAP, zero-valent iron nanoparticles (nZVI) have been identified with anticancer properties. The nZVI was originally developed to improve the magnetic properties of iron oxide-based NPs and use for the reduction of the pollutants in wastewater and environmental remediation [11, 12], biological applications such as biodiesel-producing cyanobacterium [13], and cytotoxicity effect on cancer cells [14–17]. Previous studies showed that nZVI increases ROS levels in cancer cell lines [14–16]. It causes loss of mitochondrial membrane potential and alteration in mitochondrial structure and energy metabolism [18]. Therefore, nZVI selectively kills cancer cells while being less harmful on normal cells in vitro and in vivo. This nanoparticles can excrete from the body through the liver, into bile, and into feces. In other hand, nZVI has a biodegradable nature. Also, after entering the aqueous environment and exposing, their inherent reactivity begins to decrease. Therefore, they have low toxicity and environmentally friendly nature [19–22].

Recently, several reports have been published on the effectiveness of the combined use of CAP and nanoparticles on cancer [23–28]. However, there was no study carried out to investigate the effect of nZVI and CAP on metabolic activity and apoptosis of cancer cells. Since both CAP and nZVI have a high potential to generate ROS, we hypothesized whether the combined use of these two methods might have a better anticancer effect. Therefore, we evaluated the effect of CAP and nZVI on metabolic activity of the surviving cells and apoptosis in B16-F10 melanoma cells compared to normal L929 cells.

## Materials and methods

### Ethics approval and consent to participate

The protocol of this study was approved by the Research Ethics Committee of Mazandaran University of Medical Sciences) IR.MAZUMS.REC.1398.091.)

### Chemicals and reagents

Iron (III) chloride (FeCl_3_(, sodium hydroxide, starch powder, ascorbic acid, Ethidium bromide (EtBr), and Acridine orange (AO) were purchased from Merck (Darmstadt, Germany). MTT (3-(4, 5-dimethylthiazol-2-yl)-2, 5-diphenyltetrazolium bromide) and dimethyl sulphoxide (DMSO) were purchased from Sigma (St. Louis, MO). Roswell Park Memorial Institute (RPMI)-1640, Dulbecco’s Modified Eagle’s medium (DMEM), and penicillin-streptomycin were purchased from Biowest, Germany. Fetal bovine serum and Trypsin were obtained from bioMerieux, France, and Gibco, USA. All primers were designed and purchased from Metabion, Germany. We used commercial kits for RNA extraction (Favorgen, Taiwan), cDNA synthesis (Addbio, South Korea), and Annexin V/PI apoptosis detection (BD Bioscience, New Jersey).

### Preparation and synthesis of nZVI

nZVI was prepared by reducing Fe (III) to Fe (0) using starch powder and ascorbic acid without air evacuation. The synthesis process is based on the following processes: 0.05g of starch 0.1% and 0.25g of starch 0.15% were dissolved in 50 ml of 40 g/lNaOH solution, separately. 0.81g of ascorbic acid and 0.88g of iron (III) chloride were prepared by dissolving solids in a 50 ml ethanol/water mixture with a 30/70 ratio (v/v) and stirred well. The starch 0.1% solution (0.001 M) was poured into a burette and added drop by drop into the iron chloride solution with strenuous shaking. The immediate appearance of a black color suggested the reduction of iron ions. Then 10 ml of the starch 0.15% was added such as previous step. Stirring was continued for another 20 minutes to complete the reaction. The nZVI is appeared spherical with a diameter ranging <20nm (Fig 1).

**Fig 1:** SEM image of nZVI.

### CAP device

The CAP device has consisted of a power controller, an argon gas cylinder, and a plasma jet (a cylindrical copper tube, a grounded copper ring electrode, and a Pyrex tube as a dielectric). The peak-to-peak voltage applied to the electrode was set in the range of 0–25 kV, the sinusoidal wave frequency was set to 8.8 kHz, the flow rate of argon gas (purity: 99.9999%) was 2.5 liters/min, and the distance between the nozzle and the surface of the sample solution was fixed to 30 mm. The discharge current between the metal wire (copper) and the ring electrode is 10 mA and only 5 to 10 percent of this volume is likely left from the tube, which is used for the treatment of the cells. All experiments were carried out at room temperature [29–32].

### Cell culture and viability assay

B16-F10 melanoma and L929 normal mouse cell lines were purchased from the Pasteur Institute (Tehran, Iran). B16-F10 and L929 cells were respectively cultured in RPMI-1640 and DMEM containing 10% fetal bovine serum and 1% penicillin and streptomycin. The cells were maintained in a humidified incubator at 37°C in 5% CO2 atmosphere.

MTT colorimetric assay was used to evaluate the viability of the cells [33]. In brief, 8×10^3^ B16-F10 cells/well and 1×10^4^ L929 cells/well were cultured in 96 well cell culture plates with three replications and incubated for 24 h to grow well and accommodate the new condition. Since cancerous cell line had more growth rate, we cultured a bit more normal cells in each well to equalize the number of the two cells at the time of treatment. To evaluate the effect of nZVI, the cell supernatant was exchanged with fresh media containing different concentrations (0.528–8.8 mM) of nZVI solution. To obtain the optimal effect of CAP, the cultured cells were exposed to CAP at different times (0 (untreated), 20, 30, 40, 50, and 60 s). Therefore, to evaluate the combined effect of nZVI and CAP, we used four groups: untreated, CAP, nZVI, or combined CAP and nZVI. For combination treatment, cells were first exposed to CAP and immediately treated by nZVI. In all experiments, we used IC_50_ of CAP and nZVI. After the 24h incubation, the cells received 20 μl MTT reagent (5 mg/ml in sterile phosphate-buffered saline (PBS)) and incubated at 37°C for next 4 h. Finally, the culture medium was removed and 200 μl of DMSO was added to the cells to dissolve the formazan crystals. The optical density of each well was measured at 570 nm using a microplate reader. The percentage of cell viability was calculated based on the optical density of the wells. IC_50_ was developed by an inhibition curve and recorded as the mean ± standard deviation of three independent experiments.

### EtBr/ AO staining and flow cytometric analysis for apoptosis detection

In the EtBr/ AO staining method, 8×10^3^ B16-F10 cells or 1×10^4^ L929 cells were initially seeded in a 96-well tissue culture plate and incubated for 24 h at 37°C in a humidified and 5% CO_2_ atmosphere to tolerate new condition and achieve optimal growth confluency. Subsequently, the cells were treated with CAP and/or nZVI and incubated for the next 24 h. Then, the cells were washed twice with PBS. A mixture dye consisting of 10 μl of AO (50 μg/ml) and 10 μl of EtBr (50 μg/ml) was used to stain the cells. The stained cells were visualized using an inverted fluorescent microscope in 470/40 nm at 1000 × magnification [34].

To analyze the death pattern by flow cytometry, B16-F10 and L929 cells were harvested after trypsinization, then washed in PBS and resuspended in 1x binding buffer. Annexin V-FITC and propidium iodide (PI) staining protocol was used according to the manufacturer’s recommendation. Finally, the pattern of cell death was analyzed using FloMax (Partec, Germany) [8].

### qRT-PCR

Total RNA extraction was performed according to the manufacturer’s recommendations (Favorgen, Taiwan). The expression of BAX, BCL2, and CASP3 mRNA levels were quantified using stem-loop Taqman real-time PCR assay, by unique sequence index (USI) barcodes and probe that was previously described by Fattahi et al [35]. The Glyceraldehyde-3-phosphate dehydrogenase (GAPDH) gene was used as a housekeeping gene to normalize gene expression. Primers were designed using AlleleID 6.0 software and described in our previous work [30]. To amplify the genes, we used the following thermal profile: initial denaturation at 95°C for 5 minutes followed by 40 repetitions at 95°C for 15 seconds and 60°C for 60 seconds.

### Statistical analysis

Histograms represent the mean ± SD or mean ± SE of independent experiments. Statistical analysis determined the difference between groups with normal distribution by one way of analysis of variance (ANOVA). Tukey’s post hoc test was used to perform a pair-wise comparison between groups. P-value less than 0.05 was considered significant.

## Results

### Effect of nZVI and/or CAP on the viability of the melanoma cells

As Fig 2A shows nZVI decreased the viability of the B16-F10 and L929 cells in a dose-dependent manner. However, the cytotoxic effect of nZVI on B16-F10 cells was significantly higher than on L929 cells. The optimum concentration (IC_50_) was 1.1 mM which was considered in subsequent experiments. As it was shown in Fig 2B, CAP decreased the viability of the B16-F10 cells and had no significant effect on the viability of L929 cells. A 40 s exposure to CAP was selected as the appropriate dose of CAP for subsequent experiments.

**Fig 2:** Effect of the nZVI and CAP intervention on the viability of B16-F10 melanoma and L929 normal cells. A) Different concentrations of nZVI and B) different exposure times of CAP.

The viability of the B16-F10 melanoma and L929 normal cells was determined using the MTT assay. As it was shown in Fig 3A, microscopic imaging revealed that CAP had no detrimental effect on the morphology of L929 cells compared to untreated cells. In contrast, it seems nZVI has scarcely changed the morphology of normal L929 cells. Nevertheless, CAP and/or nZVI had a significant cytotoxic effect on the B16-F10 tumor cells and caused visualized changes in the cell’s morphology. The cells were rounded and lost their connection to the bottom of the wells. In general, both treatment modalities were more effective in B16-F10 tumor cells than in L929 cells. The MTT method confirmed that the viability of B16-F10 cells was significantly reduced by CAP, nZVI, or the combined treatment compared to the untreated cells (P<0.0001) (Fig 3B). However, the effect of combined treatment on the metabolic activity of melanoma B16-F10 cells was not significantly greater than the effect of each treatment alone. Interestingly, CAP did not have a significant detrimental effect on L929 cells. However, nZVI (p = 0.018) and combined treatment (p = 0.014) showed a significant effect on L929 cells. As Fig 3B shows all treatments had a more cytotoxic effect on the B16-F10 cells when compared to the L929 normal cells (CAP (p<0.0001), nZVI (p = 0.033), and CAP/nZVI combined treatment (p = 0.015)).

**Fig 3:** The effect of CAP, nZVI, and combined of CAP and nZVI on morphological features and cell viability of B16-F10 tumor cells and L929 normal cells. A) Morphological alterations visualized under an inverted microscope (×100). B) Cell viability was assessed using the MTT method.

### Assay of apoptosis induction by AO/ EtBr staining and Annexin V-FITC/ PI flow cytometry analysis

Using fluorescence microscopy, AO staining showed that viable cells appeared uniformly green while apoptotic cells appeared red with green spots in the early stages of apoptosis and turned red with a debris nucleus in the late stage. The necrotic cells in this staining method appear uniformly red. As Fig 4 shows the CAP treatment did not affect the viability of L929 normal cells, while nZVI treatment and CAP and nVZI combination induced apoptosis and necrosis in normal cells. In the B16-F10 cancer cells, all treatments induced apoptosis and necrosis.

**Fig 4:** Apoptosis detection in B16-F10 cancer and L929 normal cells under treatment of CAP, nZVI, and combination of CAP and nZVI. A) The pattern of AO/ EtBr staining of B16-F10 cancer cell line and L929 normal cells treated using CAP, nZVI, and combination treatment. Viable cells are green in color while dead cells are red. B) Annexin V/PI flow cytometry analysis of the B16-F10 and L929 cells after harvesting by trypsinization. The graph represents the percentage of live cells, early and late apoptosis, and necrosis.

Annexin V-FITC/PI flow cytometry analysis showed that CAP did not induce apoptosis or necrosis in normal L929 cells, whereas in comparison to the untreated cells, nZVI or combined treatment with CAP and nZVI induced significant cell death in these cells. All therapeutic approaches induce cell death in the B16-F10 cells (Fig 4).

### Expression of apoptotic genes

The expression of apoptotic genes, including BAX, BCL2, and CASP3, and the ratio of BAX to BCL2 (BAX/BCL2) were assayed in melanoma cancer and normal cells using real-time PCR assay. As Fig 5 shows, all treatments changed the expression of all genes and the ratio of BAX/BCL2 ratio in B16-F10 tumor cells. On the other hand, in comparison to CAP exposure alone, CAP and nZVI combined treatment significantly increased the expression of BAX but not BCL2 and CASP3 or BAX/BCL2.

**Fig 5:** Expression of apoptotic genes in B16-F10 and L929 cells after 24 hours of CAP, nZVI, or combination therapy. Total RNA was extracted and the expression of apoptotic genes (BAX, BCL2, and Caspase-3) was evaluated by TaqMan real-time PCR. In all experiments, GAPDH was considered a housekeeping gene. Data presented as mean ± SE. The results are representative of three independent experiments.

In the L929 normal cells, CAP significantly decreased the expression of BCL2 (p<0.0001) but not BAX, CASP3, and the ratio of BAX/BCL2. nZVI and the combination therapy by CAP and nZVI significantly altered BAX, BCL2, and CASP3 expression but not BAX/BCL2 ratio.

## Discussion

In this study, we investigated the effect of combination therapy of CAP and nZVI on growth inhibition and apoptosis of melanoma cancer. It indicated CAP kills cancer cells selectivity via apoptosis and has less effect on the viability of the normal cells. The difference of ROS level between normal and cancer cells may be reason for the selectivity of CAP. Two models have been proposed to explain difference in the ROS level between the cancer and normal cells. The first model explained that tumor cells a higher baseline ROS level in comparison with normal cells. When ROS increases in the cells, total intracellular ROS in cancer cells rises above the threshold, but not in normal cells. The second model explains the existence of aquaporin (AQP) channels. These proteins transfer ROS. The cancer cells have more AQP channels and therefore, higher ROS levels (63). Our results are in line with other studies of CAP on inhibition and apoptosis in tumor cell lines [31, 36–43]. The main reason for the action of CAP is the generation of free radicals in the gas-liquid surface of the culture medium after CAP treatment and charging particles including H_2_O_2_, hydroxyl radicals (OH^−^), and singlet oxygen (•O_2_) that can self-react or interact with the medium, leading to additional RONS production. Intracellular RONS can increase caspase activity and induce apoptosis [44–49]. Because of metabolic differences between tumor and normal cells, CAP can selectively act on the tumor cells [23, 50, 51]. In other words, the plasma-free gas flow has not been shown to affect cancer cell viability but RONS produced by CAP induces a cytotoxicity activity [52, 53]. As well, in this study, nZVI induces apoptosis in cancer cells more than the normal cells. The reduced iron from nanoparticles causes oxidative stress through the production of ROS and finally causes lipid peroxidation, which leads to the loss of mitochondrial membrane potential, changes in mitochondrial structure, DNA damage and finally apoptosis [17, 18, 54].

However, this study has several limitations that should be considered when interpreting the results. In other words, cancer and normal cells were different in origin. B16-F10 is a mouse cell line with a morphology of spindle-shaped and epithelial-like cells, while L929 is a mouse fibroblast cell line. Although it is better that the target cells have the same origin, but since fibroblasts have many characteristics in the tumor microenvironment, in this study, L929 cells were used as a control, and according to ATCC® ANIMAL CELL CULTURE LINE, these cells are mouse dermal fibroblasts. These cells were widely used as normal cells in many cancer studies for comparing metabolic activity of the target cells [55–59]. Fibroblasts are the principal stromal cells that exist in the whole body and are widely distributed throughout the organs of the body such as skin. In addition, cancer-associated fibroblasts are one of the major cell content in tumor tissues. In addition, it has been reported that the usage of different condition media such as RPMI1640 and DMEM have not detrimental effect on the results [60].

We assessed the combination effect of CAP and nZVI on metabolic activity of the surviving cells and apoptosis of the B16-F10 melanoma cancer cells compared to L929 normal fibroblast cells. Several studies showed the combination of CAP and anticancer agents such as silymarin nano emulsion [8], iron oxide-based magnetic nanoparticles [24], gold nanoparticles [25], platinum nanoparticles [61], and antibody-conjugated nanoparticles [62] cause growth inhibition, induction of apoptosis and decreasing of metastasis in cancer cells. On the other hand, consistent with our findings, several studies have shown that the combined treatment of CAP and other anticancer agents such as platinum nanoparticles and curcumin has no better effect than either one alone. Removal of ROS in cells, inhibition of aquaporin channels, ROS saturation, and cell cycle arrest may explain this phenomenon [61, 63, 64]. On the other hand, our findings showed that the combination therapy had no significant improvement on toxicity compared to the nZVI or CAP alone. The cell morphological observations approved the results of the cytotoxicity test. AO/EtBr fluorescence staining and flow cytometry analysis showed that all treatments significantly induced cell death in B16-F10 melanoma cells, but the combination treatment did not have a significant additive effect compared to CAP or nZVI. The analysis of apoptosis-related gene expression, including BAX, BCL2 and CASP3, also showed that the combined treatment did not have a greater effect on the expression of apoptosis genes in cancer cells compared to CAP and nZVI alone.

Previous reports showed that BAX protein is highly expressed in malignant melanoma [65]. Other studies proved that the progression of malignant melanoma is not associated with high expression of BCL2 [66], so it is better to evaluate the BAX/BCL2 ratio in determining sensitivity to apoptotic stimuli in melanoma [67]. The results of this study showed that all treatments caused a significant increase in BAX/BCL2 ratio in B16-F10 cells compared to L929 cells. However, combined CAP and nZVI treatment did not increase the BAX/BCL2 ratio compared to CAP or nZVI alone.

Taken together, our findings demonstrated that CAP and nZVI induce more apoptosis in the B16-F10 cancer cells compared to L929 normal cells. However, combined treatment of CAP and nZVI did not increase apoptosis in B16-F10 cells compared to CAP or nZVI alone. Therefore, combination therapy of CAP and nZVI may not be more effective in inhibiting tumor growth. Several reasons may justify this event include the rate of ROS transporter into the cell having a certain capacity. When cancer cells are treated with a combination of CAP and nZVI, the further penetration of ROS into those cells is reduced due to intracellular ROS saturation [68, 69]. Transferring high concentrations of ROS into cells leads to cellular oxidation and induction of necrosis instead of apoptosis [70–73]. However, further studies are needed to prove these speculations.

## Conclusions

This study demonstrated that CAP selectively induced apoptosis in melanoma cancer cells. Also, nZVI induced apoptosis in cancer cells more than in normal cells. Combined treatment with nZVI and CAP, although it induced destruction of cancer cells, did not increase the cytotoxicity and apoptosis of B16-F10 melanoma cancer cells compared to CAP or nZVI treatment alone.

## Supporting information

S1 File MTT results of NZVI on B16-F10 and L929 cells. (PZFX)

S2 File MTT results of CAP on B16-F10 and L929 cells. (PZFX)

S3 File MTT results of CAP and NZVI on B16-F10 and L929 cells. (PZFX)

S4 File Flow cytometric analysis for apoptosis detection. (PZFX)

S5 File Expression of BAX. (PZFX)

S6 File Expression of BCL2. (PZFX)

S7 File Expression of CASP3. (PZFX)

S8 File X-ray diffraction pattern of nano particles. (DOCX)
